The article "SBAR Standard and Mind Map Combined Communication Mode Used in Emergency Department to Reduce the Value of Handover Defects and Adverse Events" was published in 2022. Journal: J Healthc Eng.

# SBAR Standard and Mind Map Combined Communication Mode Used in Emergency Department to Reduce the Value of Handover Defects and Adverse Events

**DOI:** 10.1155/2022/8475322

**Published:** 2022-03-02

**Authors:** Xiaoxuan Li, Jing Zhao, Shouzhi Fu

**Affiliations:** Emergency Department, Wuhan Third Hospital, Wuhan 430061, China

## Abstract

The objective is to explore the mind map communication mode used in the emergency department combined with the SBAR standard to reduce the occurrence of handover defects and adverse events. 180 cases of emergency treatment and patient observation from January to June 2021 were selected and studied. According to the time of admission, the selected patients were divided into observation group and control group (90 cases). The control group adopts the traditional handover mode, and the observation group thinks. The map is combined with the SBAR standard communication mode to handover; compared; and observed the two groups of nurse's handover quality scores, handover problems and adverse events, handover defects, mastery of the patient's condition and understanding of critical illness, and nursing satisfaction. The quality scores of nurses in the control group were significantly higher than those in the observation group; the incidence of adverse events in the observation group was 8.9%, and the incidence of handover problems was 2.2%, which was significantly lower than that of the control group. The mastery score of the observation group was significantly higher than that of the control group; the nursing satisfaction of the observation group was 90% significantly higher than that of the control group. The handover defect rate of 56.7% in the control group was significantly higher than that in the observation group. The nurses in the observation group had a 98.9% understanding of the critically ill patients' condition than in the control group. All the above items are statistically significant, *P* < 0.05. The combined communication mode of SBAR standard and mind map used in the emergency department can improve the quality of handover, reduce adverse events and handover problems, clear patient conditions, higher patient satisfaction, and lower handover defect rate, and nurses' critically ill patients have a higher understanding of the condition, and this communication method is worthy of clinical promotion.

## 1. Introduction

Nurse handover is an important process of transferring and obtaining information between nurses. It is generally believed that nursing errors are caused by imperfect work such as loss of patient information and work interruption during the handover process, which may affect subsequent appropriate care [1]. Therefore, it is believed that the accuracy of the nurse handover process helps to ensure the safety of patient care [2]. At present, traditional nurses often carry out collective or bedside verbal transmission, among which night nurses can carry out collective verbal transmission more frequently. This is only based on mechanical reading of the duty report, so there is a lack of reasonable control over the entire contents of the duty [3]. As a graphical tool, the biggest advantage of mind maps is that they can present complex and disordered thinking processes graphically, which is easy to understand and remember. The World Health Organization recommends using the initials SBAR. SBAR stands for [4] situation, background, assessment, and recommendation. They represent what is happening and the cause of the problem. It is the cause of the problem and how we solve the communication process. This template improves the plan by providing a template that displays patient care issues and indicates urgent issues and unfinished tasks [5]. This study explored the influence of mind map combined with SBAR standard communication mode on the quality of nurses' handover work in emergency department and achieved satisfactory results.

The article "SBAR Standard and Mind Map Combined Communication Mode Used in Emergency Department to Reduce the Value of Handover Defects and Adverse Events" was published in 2022. Journal: J Healthc Eng.

The rest of this paper is organized as follows: Section 2 discusses materials and methods, followed by the experimental results in Section 3.  Section 4 concludes the paper with summary and future research directions.

## 2. Materials and Methods

### 2.1. Clinical Data

180 patients from January to June 2021 were selected as the study subjects for emergency treatment and observation. Inclusion criteria: (1) age is 22 to 65 years old; (2) right to know the study and active participants [6]; and (3) people with relatively stable conditions in all aspects. Exclusion criteria: (1) those who have worsened conditions and need to be transferred to another department or hospital; (2) people who are unconscious or poorly communicated; (3) with severe heart, brain, kidney and other organ dysfunction; and (4) people who suffer from mental illness. This research is in line with the “Declaration of Helsinki” [7]. The selected patients were divided into the observation group (90 cases) according to the length of hospitalization (41 males, 49 females, 22–62 years old (average age is 43.69 ± 2.54 years)) and control group (54 males and 36 females, aged 23–65 years (average age is 44.21 ± 1.36)). Comparison of the general data of the two genders and age groups is not statistically significant (*P* > 0.05).

### 2.2. Methods

The control group adopts the traditional handover model, and the nurses follow the traditional handover process at the bedside, which mainly includes written materials, status information, environmental equipment, medicines, and comprehensive inspections. On the basis of the control group, the observation group uses mind mapping combined with SBAR standard communication methods. The mind map is designed according to the keyword “nurse handover,” which is mainly divided into the following three branches [8]: patient condition, ward equipment, and drug management.

1. Design a mind map, the specific thinking design is as follows. Condition [9]: mainly record the number of patients, medication, condition monitoring, psychological status, etc. Number of patients [10]: it is mainly divided into the total number of patients entering the rescue area and the observation area, the number of various levels of illness, the number of admissions and discharges, and the number of deaths. Medication [11]: pay attention to the patient's medication status, especially high-risk drugs; disease monitoring: mainly includes personal vital signs, disease diagnosis, auxiliary examinations, current treatment and nursing problems, diet and sleep, related precautions, and whether there are any security hazards, etc. Psychological status [12]: mainly focuses on whether the patient has bad emotions such as anxiety and depression, so as to prevent bad emotions from triggering suicidal thoughts and ensure the safety of patients. Condition of ward equipment: it is necessary to know the quantity of equipment in the ward and also pay attention to whether the equipment is placed in a reasonable position, whether it is disinfected, whether it is damaged, whether there is sufficient backup power supply, etc. Drug management [13]: mainly focuses on the storage, base, and expiration date of narcotic drugs, high-risk drugs, and rescue drugs.
2. Theoretical knowledge and practical training of mind mapping. The specific content includes the following [14]: specific training takes patients with sudden disease changes in the night shift as an example; for shifts caused by sudden diseases, the patients can be analyzed based on the mind map on the basis of disease monitoring. The main indicators for observing changes in the patient's condition are [15]: vital signs, complexion, physical sensation, language function, diet and excretion, skin, wounds and drainage, oxygen inhalation and ECG monitoring, and other general conditions, as well as the current main treatments, nursing and precautions, whether there is a safety hazard (risk of falling and falling from bed), and so on.

The article "SBAR Standard and Mind Map Combined Communication Mode Used in Emergency Department to Reduce the Value of Handover Defects and Adverse Events" was published in 2022. Journal: J Healthc Eng.

Specific application of mind map:

1. Formulation of the handover list: after learning the SBAR standard communication mode, under the premise of the change of the handover shift, according to the characteristics of each ward, the SBAR communication mode conversion checklist was established [16]. Based on consulting many relevant documents and visiting experts, the SBAR communication mode handover checklist was established (see Table 1).
2. SBAR training: in the SBAR nurse training, the head nurse is the core, and the nurses in this group are guided to conduct simulated situation training through specific cases. Finally, each nurse is evaluated so that each nurse has a deeper understanding and mastery of the SBAR communication mode in the nursing handover shift [17–23].
3. Handover process: before handover, nurses need to fill in the name specification. When handover, nurses need to explain the content of the shift in detail. After the handover is completed, it is necessary to repeatedly confirm whether the content of the handover is incorrect. If there are any problems, prompts should be given. Table 1 is the SBAR communication mode handover checklist in the emergency department [24].

### 2.3. Observation Indicators

Compare the shift quality of the two groups of nurses, including nurse verbal handover, bedside handover, code of conduct, and handover records; each index totals 100 points, and each item totals 25 points. Observe the adverse events that occurred in the two groups of patients, including redness and swelling at the puncture site, obstruction and shedding of the catheter, prolapse of infusion, leakage and obstruction, and disease development [25–27]. Observe the two groups of nursing staff's mastery of the patient's condition. A satisfaction survey was conducted on the two groups of nursing staff through the satisfaction questionnaire. The content of the questionnaire is mainly about the operating level, responsibility, and service attitude of the nursing staff. The score is 100 points, divided into very satisfied (over 80 points), basically satisfied (60–79 points), and dissatisfied (60 points). The defect rate of handover between the two groups of nurses mainly includes incomplete handover content, unclear pipeline retention, and incomplete handover record sheet. The two groups of nurses should consider critically ill patients. Judgment is made through a medical checklist, including basic patient information, medical conditions, examination results, and treatment points. Each project is divided into three options: complete understanding, partial understanding, and not understanding, using SPSS 20 software for data processing. Data counts are expressed by instance, percentage, and chi-square test; measured data are expressed by $\bar{x}\pm s$ and pass the *t*-test. The difference of *P* < 0.05 is statistically significant.

The article "SBAR Standard and Mind Map Combined Communication Mode Used in Emergency Department to Reduce the Value of Handover Defects and Adverse Events" was published in 2022. Journal: J Healthc Eng.

## 3. Clinical Data and Analysis

### 3.1. Comparison of Handover Quality Scores between the Two Groups of Nurses

The scores of nurses in the control group for oral shift (24.36 ± 1.96), bedside handover (24.96 ± 1.36), code of conduct (24.13 ± 1.69), and shift record (23.39 ± 1.55) were significantly higher than those of the observation group (21.46 ± 3.24), bedside handover (19.56 ± 3.85), code of conduct (22.36 ± 2.69), and shift record (20.69 ± 2.56).  Table 2 shows the comparison of handover quality scores of the two groups of nurses.

### 3.2. Comparison of Adverse Events and Handover Problems between the Two Groups of Patients

The incidence of adverse events in the observation group was 8.9%, and the incidence of handover problems was 2.2%, which was significantly less than the 23.3% of adverse events in the control group and 18.9% of handover problems. The difference was statistically significant (*P* < 0.05).  Table 3 displays comparison of adverse events and handover problems between the two groups of patients.

### 3.3. Comparison of Nurses' Knowledge of the Two Groups of Patients

The mastery score of the observation group was significantly higher than that of the control group. The reason for hospitalization was 9.34 ± 0.13, the past history was 9.63 ± 0.35, the difference in auxiliary examination of disease changes was 9.19 ± 0.36, the treatment and nursing methods were 9.21 ± 0.34, the potential risk was 9.07 ± 0.55, and the key point of nursing was 9.64 ± 0.25, and all mastery scoring items are statistically significant (*P* < 0.05).  Table 4 shows comparison of nurses' knowledge of the two groups of patients.

### 3.4. Comparison of Patient Care Satisfaction between the Two Groups

The nursing satisfaction rate of the observation group was 90% significantly higher than that of the control group 64.4%, and the difference was statistically significant (*P* < 0.05).  Table 5 is the comparison of nursing satisfaction between the two groups of patients.

### 3.5. Comparison of Deficiencies in Handover between the Two Groups

The handover defects of the two groups included incomplete handover content, unclear pipeline retention, and incomplete handover records. The handover defect rate of the control group was 56.7% significantly higher than that of the observation group 11.1%, and the difference was statistically significant at *P* < 0.05.  Table 6 is the comparison of deficiencies in handover between the two groups.

### 3.6. Comparison of the Understanding of Critically Ill Patients between the Two Groups of Nurses

One month after nursing in the observation group, the nurses' understanding of the critically ill patients' condition was higher than that of the control group. The total understanding rate of the observation group was 98.9%, and the total understanding rate of the control group was 92.3%. The difference of *P* < 0.05 was statistically significant.  Table 7 shows the comparison of the understanding of critically ill patients between the two groups of nurses.

The article "SBAR Standard and Mind Map Combined Communication Mode Used in Emergency Department to Reduce the Value of Handover Defects and Adverse Events" was published in 2022. Journal: J Healthc Eng.

After using the SBAR communication model in my nursing handover shift, the nurses' understanding of the patient's condition has improved, which has effectively reduced the risk of adverse nursing events. After the SBAR communication mode is used to change the nursing shift, nursing professionals can quickly understand the key points of patient care and facilitate the development of high-quality personalized biochemical nursing services for patients. The long-term use of SBAR communication mode for referral work has improved the nurses' ability to simultaneously assess and identify the patient's condition and help improve the nurse's comprehensive nursing ability. At the same time, the teamwork ability of nurses has also been effectively improved.

## 4. Conclusion

Although the shift time is short, the morning shift reflects the comprehensive quality and management level of the nurses in the ward. Accurate and concise handover is the beginning of the day's work. Therefore, the “SBAR mode morning shift report form” is adopted for shift. The SBAR communication mode can provide nurses with instant and accurate nursing information, and the efficiency of nursing information transfer between nurses is higher. Using SBAR communication mode to transfer nursing work, the information transmission between nurses is more systematic, which can effectively avoid the chaotic spread of information and greatly improve the overall work efficiency of the medical team. The SBAR communication mode is applied to the field of first aid, which can effectively shorten the rescue preparation time and improve the rescue efficiency, which is of great significance to saving the lives of patients.

This paper uses SBAR standards and mind map communication mode for emergency services, which can improve the quality of referrals, reduce bad cases and referral problems, understand the patient's condition more clearly, improve patient care satisfaction, and reduce the referral rate. It is worthy of clinical promotion.

## Figures and Tables

**Table 1:** SBAR communication mode handover checklist in the emergency department.

Date/time		
S	Current situation	Bed number
		Name
		Age
B	Backgrounds	Past history
		Allergies
		Diagnosis
		Symptom
		Physical signs
		Awareness
		Pupil
		Vital signs
A	Evaluation	Pipeline situation
		Skin condition
		Medical treatment
R	Suggestion	Guiding advice
		Unresolved issues
		Unfinished task

The article "SBAR Standard and Mind Map Combined Communication Mode Used in Emergency Department to Reduce the Value of Handover Defects and Adverse Events" was published in 2022. Journal: J Healthc Eng.

**Table 2:** Comparison of handover quality scores of the two groups of nurses.

Group	Oral handover	Bedside handover	Code of conduct	Handover record
Control group	21.46 ± 3.24	19.56 ± 3.85	22.36 ± 2.69	20.69 ± 2.56
Test group	24.36 ± 1.96	24.96 ± 1.36	24.13 ± 1.69	23.39 ± 1.55
*T*	3.010	4.640	3.226	4.522
*P*	0.006	0.000	0.002	0.000

**Table 3:** Comparison of adverse events and handover problems between the two groups of patients (%).

Group	*n*	Adverse events	Handover problems
Control group	90	21 (23.3)	17 (18.9)
Test group	90	8 (8.9)	2 (2.2)

**Table 4:** Comparison of nurses' knowledge of the two groups of patients.

Group	*n*	Reason for hospitalization	Past history	Auxiliary examination of changes in condition	Treatment and care methods	Potential risks	Key points of care
Control group	90	7.15 ± 0.45	7.48 ± 0.39	6.47 ± 0.57	7.95 ± 0.48	7.38 ± 0.33	7.29 ± 0.37
Test group	90	9.34 ± 0.13	9.63 ± 0.35	9.19 ± 0.36	9.21 ± 0.34	9.07 ± 0.55	9.64 ± 0.25

**Table 5:** Comparison of nursing satisfaction between the two groups of patients.

Group	*n*	Very satisfied	Basically satisfied	Dissatisfied	Total satisfaction %
Control group	90	38	20	32	64.4
Test group	90	56	25	9	90

**Table 6:** Comparison of deficiencies in handover between the two groups.

Group	*n*	The content of the handover is not comprehensive (case %)	The pipeline retention situation is not clear (case %)	Incomplete transfer records (example %)	Defect rate (%)
Control group	90	5 (5.6)	2 (2.2)	3 (3.3)	11.1
Test group	90	17 (18.9)	16 (17.8)	18 (20)	56.7
*X* ^2^					18.442
*P*					0.002

**Table 7:** Comparison of the understanding of critically ill patients between the two groups of nurses.

Group	*n*	Fully understand	Partial understanding	Incomprehension
Control group	90	87 (96.7)	2 (2.2)	1 (1.1)
Test group	90	51 (56.7)	32 (35.6)	7 (7.8)
*X* ^2^		6.856	5.741	4.569
*P*		0.042	0.051	0.048

## Data Availability

The data used to support the findings of this study are available from the author upon request.
